# Evaluation of Bacterial Cellulose Dressing versus Vaseline Gauze in Partial Thickness Burn Wounds and Skin Graft Donor Sites: A Two-Center Randomized Controlled Clinical Study

**DOI:** 10.1155/2022/5217617

**Published:** 2022-05-18

**Authors:** Xuanliang Pan, Chunmao Han, Guoxian Chen, Youfen Fan

**Affiliations:** ^1^Department of Burns and Wound Repair, The Second Affiliated Hospital of Zhejiang University School of Medicine, Hangzhou 310009, Zhejiang Province, China; ^2^Burn Care Center, Hwa Mei Hospital, University of Chinese Academy of Sciences, Ningbo, China

## Abstract

**Objective:**

Bacterial cellulose (BC) dressing, which can maintain a moist environment and prevent the invasion of pathogens, has become a competitive dressing material for burn wound treatment. This study was conducted to evaluate the treatment efficacy of a novel China-made BC dressing for the treatment of second-degree burn wounds and skin graft donor sites.

**Methods:**

212 patients with second-degree burn wounds or skin graft donor sites were enrolled from two research centers. They were randomly assigned to the BC dressing group (study group) or the Vaseline gauze (VG) dressing group (control group). Wound conditions were assessed before and after treatment. Dressings were changed according to the condition of the wound bed. Healing rate and healing time were recorded as primary endpoints to evaluate the efficacy of BC dressing against VG dressing. Erythema, swelling, exudation, bleeding, subeschar purulence, and pain were assessed as secondary endpoints.

**Results:**

207 participants completed the trial and their wounds all healed within 28 days. The average healing times for superficial and deep secondary burn wounds and skin graft donor sites in the BC group were 8.12, 15.77, and 10.55 days, respectively. In the VG group, the average healing times for superficial and deep secondary burn wounds and skin graft donor sites were 9.30, 15.27, and 11.19 days, respectively. The healing time of superficial burn wounds in the BC group was statistically shorter than that in the VG group. There was no difference in the frequency of dressing changing between two groups. The BC dressing showed equal efficacy with the VG dressing at all secondary endpoints.

**Conclusion:**

The novel BC dressing could be used for the management of second-degree burn wounds and skin graft donor sites. With a shorter healing time in superficial secondary burn wound than that of the VG dressing, the BC dressing showed noninferiority in the treatment of superficial and deep secondary burn wounds and skin graft donor sites versus the VG dressing. This study is registered with the Chinese Clinical Trial Registry (registry number: ChiCTR1800014377 (http://www.chictr.org.cn)).

## 1. Introduction

Burn wound due to thermal injury is one of the public health problems in modern society, usually causing irreparable harms and a variety of side effects for victims and their families. Generally, burn wounds are classified into 3 categories according to their severity or the depth of the tissues affected [1] Among them, second-degree (partial thickness) burns feature blisters covering a red base and the lesion reaches the deep skin layers, which is further classified into superficial and deep partial thickness burns. The depth of the burns directly affects the healing and scarring of the wounds [2].

The healing of second-degree burn wounds is a complex process that depends on the tissues, cell types, and matrix components [3]. Thus, the management of second-degree burns is still controversial [4]. Without the protection of the integumentary system, the burn wound bed is under high risk of bacterial infection, disrupting the natural healing process and leading to poor outcomes. Therefore, wound dressings that can maintain a moist environment and prevent the invasion of pathogens are of great importance to the treatment of second-degree burns [5]. Clinically effective wound dressings should also possess the features of excellent water retention capacity, ideal biocompatibility, comfort for the patients, and ease of application [6].

A wide variety of dressing materials, such as honey, silver sulfadiazine dressing, and chitosan, have been tested for the treatment of second-degree burn wounds [7, 8]. However, due to adherence to the wound surface, personal suffering in dressing change, and delayed healing, few of them have been well approved [9]. Bacterial cellulose (BC) is natural cellulose fermented from *Acetobacter xylinum* and other bacteria. Due to high purity and the absence of some typical plant components such as lignin, pectin, and hemicelluloses, BC is considered as a noncytotoxic and highly biocompatible material with several desirable characteristics, such as high permeability, absorbability, wet tensile strength, flexibility, elasticity, and biocompatibility. Today, BC is being actively investigated and developed as both an independent and composite dressing material for the treatment of burn wounds [10, 11]. With the optimization of interconnection of the fibers and nanosized pore structure, some novel BC can even be used as an antimicrobial wound dressing with a desirable sustained release functionality for targeting persistent bacterial pathogens [6]. Assembling the silver nanoparticles on the surface of BC has attracted increasing attention and has become an effective strategy of developing burn wound dressing with antibacterial property [12, 13]. However, accumulating evidence suggests that chemical contaminations may be induced during the functionalization of BC [14]. Exposure of the burn wounds to silver ions or compounds may delay the reepithelialization of wounds due to the significant cytotoxicity [15]. In the light of safety, biocompatibility, and cost, these randomized controlled trials (RCTs) were conducted to investigate the treatment efficacy of a novel BC in its original form as a dressing for second-degree burn wounds and skin graft donor sites. Vaseline gauze (VG) dressing was used as the control.

## 2. Materials and Methods

### 2.1. Patients

Since January 2018, consecutive patients of both sexes with second-degree burns who have been presenting at the Second Affiliated Hospital of Zhejiang University School of Medicine and Ningbo No. 2 Hospital were screened for the eligibility of this study. The inclusion criteria were as follows: (1) being aged 18 to 65 years, (2) being diagnosed with second-degree burns or partial-thickness skin graft donor wound within 24 hours of admission, and (3) burn wound bed area larger than 100 cm^2^ but less than 15% of total body surface area (TBSA) [16]. Patients with the following features were excluded: (1) impaired cardiovascular function (signs and symptoms of cardiac failure), (2) impaired hepatic function (serum total bilirubin was 1.5 times higher than the upper limit of normal value), (3) impaired renal function (increased blood creatinine and urea nitrogen), (4) hematological complications, (5) severe hypoalbuminemia (plasma albumin <25 g/L), (6) severe systemic infection (e.g., septicemia), (7) uncontrolled diabetes mellitus, (8) use of corticosteroids, (9) pregnancy or breast-feeding, (10) participation in other clinical trials three months prior, and (11) skin disorder, allergic disorder, or other conditions that could interfere in the study assessment. All eligible participants could leave the clinical trial at any time for any reason. Participants who did not complete the clinical trial were considered dropouts.

The present clinical trial was approved by the Ethics Committees of the Second Affiliated Hospital of Zhejiang University School of Medicine. Written informed consent was acquired from all the participants. The study was carried out in accordance with the Declaration of Helsinki. Demographic and clinical data were properly collected and protected by all investigators.

### 2.2. Sample Size and Randomization

This was a noninferiority trial [17], intended to prove that the efficacy of BC dressing was not inferior to that of the VG dressing in the management of second-degree burn wounds or partial-thickness skin graft donor sites. Hence, the ratio of participants between the two treatments was predetermined as 1:1. The sample size was estimated according to the statistical significance (*α* = 0.05, *β* = 0.2) reported previously [16], and the dropout rate (6%) and the treatment efficacy (90%) were predetermined by our preliminary data. The random allocation of patients was conducted as per the random number generated by computer program. A total of 212 patients were enrolled and randomly assigned into two BC and VG dressing groups, with 106 participants for each group. Only one wound was observed in each participant. The process of enrollment and randomization is shown in Figure 1.

### 2.3. BC and VG Dressing

The BC dressing material tested was produced by Shenzhen Ai Jie Te Medical & Pharmaceutical Science and Technology LLC (Shenzhen, China). As commercial secrets, the recipe, production, and specifications of the BC dressing material are not disclosed here. The BC dressing had passed vigorous quality tests before being used in this clinical trial. The typical BC dressing measured 20 cm × 20 cm. VG dressing is widely used in clinical practice for the management of burn wounds as well as a control in clinical trials. It was prepared as reported previously [18]. Both BC dressing and VG dressing were tailored to fit the size and shape of the wounds in each participant.

### 2.4. Clinical Treatment and Evaluation

The area of a wound was measured with a disposable piece of transparent plastic with 1 cm × 1 cm grids printed on it. A marker was used to trace the boundary of the wound on the plastic. The number of grids within the boundary was used to calculate the area.

The burn wounds were cleaned with normal saline before being treated with either the BC or the VG dressing according to the randomized grouping. The donor sites were covered immediately after skin harvesting. A sterile gauze pad, covering the BC or VG dressing, was typically changed once every two days. If excessive volume of exudate was observed, the sterile gauze pad was changed on a daily basis. BC and VG dressings were not changed periodically. Instead, they were only changed according to the conditions of wounds. If the adherence between the dressing and a wound bed was strong and no collection of exudates was observed, the dressing remained in place until the wound healed. Otherwise, an opening was made to drain the exudate and the dressing was changed at the doctor's discretion.

The healing process, the conditions of the wound bed, and the changes of dressing were carefully observed and recorded until the end of the trial on day 28 of treatment. For wounds that healed completely, the time taken for complete healing was recorded. For wounds that failed to heal completely within the 28 days, the leftover area of the wound bed was measured to calculate the percentage of the wound that healed.

A wound bed area of 100 cm^2^ was selected from each participant. The primary endpoints were wound bed healing rate (WBHR) and the time for complete wound healing. The healing rate was calculated as previously described [19]. Standards for evaluation of efficacy are listed in Table 1.

A scoring method consisting of four components was developed to characterize the conditions of wounds. The components are erythema and swelling, exudation, hemorrhage, and subeschar purulence and exudation. The score of each component ranges from 1 to 4, representing the increasing severity of the condition of a wound (Table 2).

The pain caused by the burn wounds was assessed according to the visual analogue scale (VAS) [20]. Pain was considered as severe for a score of 6–10, moderate for a score of 4-5, mild for a score of 2-3, and relieved for a score of 0-1. Data of adverse events was collected per International Committee for Harmonization guidelines for Good Clinical Practice as described previously [21]. Demographic data and the results of necessary clinical tests were filed individually.

Blood and urine samples were analyzed for screening of eligibility of the patients based on inclusion and exclusion criteria. Cardiovascular, hepatic, and renal functions were monitored during the hospitalization of each participant as a routine of our clinical practice.

### 2.5. Statistical Analysis

The difference in appearance between a BC dressing and a VG dressing was obvious. Hence, blinding was not applicable for both the participants and the clinical workers. To alleviate possible biases, the estimation of sample size [16], random allocation of patients [22], and statistical analysis of this study were performed by a third party, the Department of Epidemiology and Health Statistics, Wuhan University School of Health Sciences, Wuhan, China.

EpiData software (version 3.0, Odense, Denmark) was used for data entry and verification. SAS (version 9.1.3, Cary, NC) was used for the statistical analysis. Data were presented as mean ± SD, median (range) or frequency (*n*/*n*), or percentage (%). The difference between the two groups was analyzed by Student's *t*-test, chi-squared test, Fisher's Exact Test, or Mann–Whitney *U* test where appropriate. A *p* value less than 0.05 was considered statistically significant. All tests were two-tailed unless otherwise stated.

## 3. Results

### 3.1. Characteristics of the Participants

248 patients were screened for their eligibility for this clinical trial. Among them, 36 patients were excluded due to age, pregnancy, breast-feeding, or other conditions (Figure 1). In total, 212 patients were enrolled in this trial. In the BC group, 4 participants dropped out from the cohort: 1 participant who changed her mind, 2 who transferred to other hospitals, and 1 who did not like to be treated with BC. In the VG group, only 1 participant gave up treatment due to financial reasons. Therefore, only 5 participants dropped out from the study, yielding a dropout rate of 2.4%, less than the preset value (6%) for the estimation of sample size. Hence, we contend that the sample size is satisfactory for this clinical trial.

The average ages of the participants in the BC and VG groups were 42 and 45 years, respectively, with no statistically significant differences found (*p*=0.137). In this study, the incidence rate of second-degree burns in the middle-aged group was much higher than that of other age groups. The proportions of participants with a history of allergy in the two cohorts were as low as 5.88% and 5.71%, respectively. No difference was observed in the history of allergy, comorbidity, blood pressure, heart rate, and breath rate, indicating that the cohorts for the BC treatment and the VG treatment were comparable (Table 3).

Ninety-six participants were diagnosed with superficial second-degree burn wounds, while only 24 patients suffered from deep second-degree burn wounds. All body parts were at risk of being burned. However, the right lower limb was the most frequently (31.88%) injured body part, followed by the left lower limb, with a much lower incidence rate of 18.84% than the former (Table 4). No statistical difference was observed regarding the age, education level, marriage, history of allergy, type of wounds, and the location of wounds between the two groups, which suggests that the patients in the two cohorts were comparable.

Major laboratory test results are shown in Table 5. No statistically significant difference was found between the two groups either before or after the treatment. However, some of the parameters such as the count of white blood cells (WBC) and platelet (PLT), the concentration of hemoglobin (Hb), and total bilirubin (TBIL) improved after treatment in both groups.

### 3.2. Healing Effect of BC Dressing

Both BC dressing and VG dressing showed high efficacy in the management of burn wounds and skin graft donor sites; all wounds healed within 28 days. The healing time for different wound types was variable. In both groups, the healing time for superficial wounds was the shortest, followed by that of skin graft donor sites, at about 11 days. Deep second-degree wounds took the longest time to heal, about 15 days (Table 6). It is worth noting that the average healing time of superficial wounds in BC group was more than one day shorter than that of VG group (*p*=0.029).

The frequencies of dressing changing in different wound types were variable. However, no difference was observed in the two groups. The BC dressing was flexible and translucent, which made it easier for doctors and nurses to observe the wound and make suitable discretion regarding the changing of dressing and alleviate unnecessary pain in patients (Figure 2). Adverse events were observed in 5 participants in the BC group, while 11 cases were reported in the VG group. The signs of adverse events included rashes, increased alanine aminotransferase (ALT) and total bilirubin (TBIL), decreased albumin, and urine occult blood. These adverse events were promptly and successfully resolved without disrupting the treatment process.

Wound conditions and healing process were assessed from four aspects: erythema and swelling, exudation, bleeding, and subeschar purulence and exudation. Wound conditions before treatment are listed in Table 4. Erythema and swelling presented in all wounds and were mostly mild and moderate. Wound exudation was also a significant symptom in all participants; about 22% of the participants even suffered from severe wound exudation. Around 44% of the participants in the BC group did not suffer from would bleeding, while in the VG group, only 35% did not. No difference was found regarding the bleeding in the two groups before treatment (*p*=0.264). In both groups, only a small proportion of the participants experienced subeschar purulence and exudation. The score of the wound conditions before and after the treatment and the comparison between the two treatment groups are shown in Table 6.

BC dressing was very helpful for the reepithelialization of wounds. From day 3 to day 7, the changes in the erythema, swelling, exudation, and bleeding were statistically significant. The score of subeschar purulence remained very low in the BC group throughout the whole process of treatment. Hence, it is reasonable to infer that the changes in subeschar purulence were not statistically significant. BC dressing was also good at pain relieving. The pain score in the BC group decreased quickly and significantly within 7 days of treatment and remained at a very low level until the healing of the wounds (Table 7).

## 4. Discussion

Results collected from well-conducted randomized controlled trials (RCTs) are regarded as top-tier evidence for decision-making in clinical practice [23], which has been used to compare the efficacy between novel, conventional, and commercial dressings for burn wounds [24, 25]. The present RCT was a prospective, comparative, quantitative clinical study conducted under controlled conditions with random allocation of treatments to comparison groups. Additionally, this study was implemented in accordance with the guidance of SPIRIT (Standard Protocol Items: Recommendations for Interventional Trials) [26]. To ensure the reliability of this study and eliminate possible confounding factors, the design and implementation of the study and the data analysis and interpretation of findings were carefully performed to assess the effect of the treatment and how far it deviated from its true value. For instance, the study was conducted in two hospitals that have similar research teams but are located in different cities. In this scenario, the participants were allocated into two independent research centers rather than single center, helpful for controlling selection and observer biases [27]. Blinding is a good strategy to alleviate introducing unconscious information bias to the participants and/or the investigators. Therefore, the study design and vigorous statistical analysis were performed by a third party with proper statistical methods. In addition, the dropout rate of this study was only 2.4%, less than the preset value of 6%. Thus, we are confident with the results and the power of this RCT.

The treatment of partial thickness burn wounds is healing-effect-oriented. The advances in material sciences have deepened understanding of wound healing and infections and driven the development of new dressings [28]. Today, a wide variety of dressings are available in the market or have been tested in clinical practice [5, 29]. The materials used for dressing include hydrocolloid, polyurethane film, hydrogel, silicon-coated nylon, biosynthetic skin substitute, antimicrobial, fiber, and pads [30]. It is well known that the treatment of second-degree burn wounds is very challenging due to significant fluid loss, repeated and painful dressing changes, and wound infection, leading to local tissue damage and complications. Due to the lack of high-quality evidence collected from RCTs, it is still risky to confirm the healing effect of a specific dressing on the treatment of second-degree burn wounds [31].

VG dressing has been used widely for the treatment of second-degree burn wounds or skin graft donor sites in clinical setting and as a reference for the evaluation of new dressing materials [18, 32–34]. BC has many intrinsic characteristics; it is nontoxic and biocompatible, and its high capacity of water retention makes it an ideal material for burn wound dressing [9]. In the present RCT, we evaluated the efficacy of a novel BC dressing against VG dressing. Based on our observation, the novel BC dressing demonstrated the following desirable characteristics: (1) It was elastic and could accommodate necessary movements of the participants. (2) It was adhesive and could conform to the wound bed perfectly, protecting the wound from infections. (3) With the reticulate structure of thin fibers coupled with superior water retention capacity [35], it could absorb exudate and maintain moisture of the wound and facilitate oxygen exchange as well, accelerating reepithelialization for burn wounds. According to the results (Table 7), with the treatment of BC dressing, the four components of the scoring method, erythema and swelling, exudate, hemorrhage, and subeschar purulence and exudation were well controlled. They disappeared within 7 days of treatment, leading to a healing rate of 100% in 28 days.

Compared to VG dressing, the average healing time of BC dressing treatment for superficial wound was about 1 day shorter (*p*=0.029). However, the healing times in deep wounds and skin graft donor sites of BC dressing were the same as those of the VG group. The difference in healing time of BC dressing may be because of the characteristics that were covered previously [9, 35]. However, bench-scale studies, well-designed animal experiments, and clinical trials with larger sample sizes are required to explore possible mechanism. The healing time of this study was much shorter than those in some previous reports. The efficacies of Nitrofurazone, Vaseline gauze, and ColActive Plus Ag were compared in an RCT for a wound bed with an area of about 45 cm^2^, which is much smaller than the area observed in this study. However, it took more than 12 days for superficial burn wounds to heal in the previous study [18]. In other RCTs, VG was used as a control to compare the efficacies of other dressings, and the healing time was longer and the healing rate was lower than in this study [32, 33].

The changing of dressings in patients with burn wounds is time-consuming. It might take 105 minutes to dress a facial burn wound and 66 minutes to change a dressing on a hand [9]. In this study, as the differences between BC and VG dressings were obvious, it was difficult to evaluate the time consumed on dressing changing objectively. Therefore, the time consumption of dressing changing was not compared. In addition, the BC dressing tested in this study was produced on a small scale for the clinical trial. Its cost was much higher than that of the VG dressing. Therefore, the cost effectiveness of the two dressings was not compared. It is arguable that when the BC dressing becomes produced on a commercial scale, its cost effectiveness will be close to that of VG dressing.

Despite the aforementioned advantages, this RCT has some limitations. Due to careful ethical considerations, the wound bed area of each participant was strictly controlled to less than 15% of the total body surface area (TBSA) and only one wound bed was observed in each participant. Limited treating area may affect the generalization and extrapolation of the findings of this study. To compare the treatment efficacies of BC dressing and VG dressing, a set of primary and secondary endpoints were observed. However, as two of the major impact factors on burn wound healing, the etiology and severity of wound infections and the response of host were not included.

In the future, a multicentered study with a much larger sample size should lead to better conclusions. For greater effectiveness, if ethically possible, the BC dressing and control dressing, such as hydrocolloids and hydrofiber dressing scan, be applied on the same participant simultaneously, though it may affect the measurement of pain and tolerance level when a normal visual analogue score scale is used.

## 5. Conclusions

The results of this noninferiority trial demonstrated that the novel BC dressing could be used for the management of second-degree burn wounds and skin graft donor sites. The BC dressing was superior to the VG dressing in the treatment of superficial second-degree burn wounds in terms of healing time. The BC dressing also showed noninferiority in the management of deep secondary burn wounds and skin graft donor sites versus VG dressing. The tested novel BC dressing has vast potential for future application in clinical practice.

## Figures and Tables

**Figure 1:** The flowchart of the randomized controlled clinical trial on wound dressing.

**Figure 2:** The application of BC dressing and VG dressing in second-degree burn wounds. Bacterial cellulose (BC) dressing and Vaseline gauze (VG) dressing were used in second-degree burn wounds in the two-center randomized controlled clinical study. Their treatment efficacies were compared as well. (a) Deep second-degree burn wound on left forearm. (b) BC dressing was applied. BC dressing was translucent, which allowed the wound to be checked easily. (c) Without changing BC dressing, wound healed on day 12; BC dressing dried up and fell off. (d) Deep second-degree burn wound on right forearm. (e) VG dressing was less translucent than BC dressing, making checking less convenient. 12 days later, VG was stuck to the wound bed and was not able to be changed. Hemorrhage was observed when changing outer cover of VG. (f) Wound healed on day 21, but there were difficulties when removing VG.

**Table 1:** Standards for evaluation of treatment.

WBHR	Evaluation
WBHR = 100%	Complete healing
50% ≤ WBHR < 100%	Significant effectiveness
20% ≤ WBHR < 50%,	Effectiveness
WBHR < 20%	Ineffectiveness

Note: WBHR, wound bed healing rate.

**Table 2:** The scoring method for evaluation of wound conditions.

Wound condition	Score
No sign	1
Mild sign	2
Moderate sign	3
Sever sign	4

**Table 3:** Demographic and clinical baseline information of the participants.

Variable	BC group (*n* = 102)	VG group (*n* = 105)	*p* value
Age			
18-	14 (13.72)	12 (11.43)	0.137
28-	30 (29.41)	17 (16.19)	
38-	27 (26.47)	37 (35.24)	
48-	23 (22.55)	31 (29.52)	
58–65	8 (7.85)	8 (7.62)	
Education			
Primary school	28 (27.45)	30 (28.57)	0.105
Middle school	43 (42.16)	57 (54.29)	
High school	17 (16.67)	16 (15.24)	
College and above	14 (13.72)	2 (1.90)	
Marriage			
No	17 (16.67)	13 (12.38)	0.381
Yes	85 (83.33)	92 (87.62)	
Systolic BP (mm Hg)	129.52 ± 17.58	132.87 ± 17.52	0.173
Diastolic BP (mm Hg)	77.98 ± 12.46	81.01 ± 14.67	0.112
Breath rate (per min)	19.22 ± 1.29	19.16 ± 1.57	0.789
Heart rate (per min)	83.51 ± 10.97	82.08 ± 12.54	0.383
History of allergy			
No (%)	96 (94.12)	99 (94.29)	0.959
Yes (%)	6 (5.88)	6 (5.71)	
Comorbidity			
No (%)	96 (94.12)	98 (93.33)	0.816
Yes (%)	6 (5.88)	7 (6.67)	

**Table 4:** Characteristics of the wounds in participants.

Variable	BC group (*n* = 102)	VG group (*n* = 105)	*p* value
Wound type			
Superficial II° burn	49 (48.04)	47 (44.76)	0.695
Deep II° burn	13 (12.74)	11 (10.48)	
Skin graft donor	40 (39.22)	47 (44.76)	
Wound location			
Trunk	13 (12.75)	14 (13.33)	0.586
Right upper limb	8 (7.84)	11 (10.48)	
Right lower limb	31 (30.39)	35 (33.33)	
Left upper limb	13 (12.75)	9 (8.57)	
Left lower limb	23 (22.55)	16 (15.24)	
Craniofacial region	14 (13.72)	19 (18.10)	
Bilateral upper limb	0 (0.00)	1 (0.95)	
Erythema and swelling			
None	14 (13.73)	16 (15.24)	0.539
Mild	39 (38.24)	42 (40.00)	
Moderate	33 (32.35)	34 (32.38)	
Severe	16 (15.68)	13 (12.38)	
Exudate			
None	1 (0.98)	0 (0.00)	0.503
Mild	33 (32.35)	29 (27.62)	
Moderate	46 (45.10)	53 (50.48)	
Severe	22 (21.57)	23 (21.90)	
Hemorrhage			
None	45 (44.12)	37 (35.24)	0.264
Mild	39 (38.24)	47 (44.76)	
Moderate	14 (13.72)	18 (17.14)	
Severe	4 (3.92)	3 (2.86)	
Subeschar purulence and exudation			
None	89 (87.25)	98 (93.33)	0.136
Mild	12 (11.77)	7 (6.67)	
Moderate	0 (0.00)	0 (0.00)	
Severe	1 (0.98)	0 (0.00)	

**Table 5:** Blood and urine test results of the participants.

Parameter	BC		VG		*p* value			
	Before (*n* = 102)	After (*n* = 102)	Before (*n* = 105)	After(*n* = 105)	BC (beforeversus after)	VG (beforeversus after)	BC versusVG (before)	BC versusVG (after)
WBC (10^9^/L)	11.00 ± 5.75	8.43 ± 3.91	10.37 ± 4.21	9.03 ± 3.95	0.01	0.018	0.362	0.273
RBC (10^12^/L)	5.17 ± 4.34	4.34 ± 0.66	4.72 ± 1.99	4.48 ± 2.02	0.058	0.398	0.332	0.508
Hb (g/L)	143.07 ± 20.29	131.02 ± 19.33	135.82 ± 22.89	128.53 ± 19.90	0.01	0.015	0.017	0.363
PLT (10^9^/L)	228.40 ± 100.30	306.27 ± 109.03	252.16 ± 110.28	314.80 ± 119.72	0.01	0.01	0.107	0.593
ALT (U/L)	35.85 ± 45.64	47.29 ± 51.09	29.15 ± 22.38	44.91 ± 53.98	0.093	0.006	0.179	0.746
AST (U/L)	36.33 ± 56.52	30.07 ± 25.18	33.62 ± 67.45	28.19 ± 22.76	0.308	0.438	0.754	0.575
Albumin (g/L)	35.61 ± 6.39	37.10 ± 6.09	35.14 ± 6.56	36.66 ± 6.88	0.090	0.104	0.605	0.628
TBIL (*μ*M)	14.34 ± 6.30	8.95 ± 4.19	13.04 ± 7.50	9.50 ± 5.57	0.01	0.01	0.183	0.427
BUN (mM)	4.81 ± 3.35	4.34 ± 1.40	5.22 ± 6.67	4.23 ± 1.41	0.192	0.138	0.573	0.592
Creatinine (*μ*M)	65.75 ± 16.56	62.21 ± 13.95	61.38 ± 13.62	59.04 ± 16.86	0.100	0.271	0.039	0.143
Uric acid (*μ*M)	260.82 ± 97.62	258.52 ± 94.44	262.86 ± 85.75	266.42 ± 93.97	0.865	0.777	0.874	0.533
Proteinuria	28 (27.45)	23 (22.55)	29 (27.62)	18 (17.14)	0.419	0.069	0.982	0.329
WBC in urine	23 (22.55)	7 (6.86)	17 (16.19)	8 (7.62)	0.002	0.055	0.243	0.834
RBC in urine	26 (25.49)	13 (12.74)	21 (20.00)	16 (15.24)	0.014	0.365	0.339	0.605

Note: WBC, white blood cell; RBC, red blood cell; Hb, hemoglobin; PLT, platelet; ALT, alanine aminotransferase; AST, aspartate aminotransferase; BUN, blood urine nitrogen; TBIL, total bilirubin.

**Table 6:** Treatment efficacy of BC and VG dressings in partial-thickness burn wounds and donor sites.

Variable	BC group			VG group			*p* value		
	Superficial II° wound (*n* = 49)	Deep II° wound (*n* = 13)	Donor site (*n* = 40)	Superficial II° wound (*n* = 47)	Deep II° wound (*n* = 11)	Donor site (*n* = 47)	Superficial II° wound	Deep II° wound	Donor site
Healing time (day)	8.12 ± 2.15	15.77 ± 5.04	10.55 ± 4.40	9.30 ± 3.68	15.27 ± 5.27	11.19 ± 3.88	0.029	0.408	0.236
Healing rate (%)	100	100	100	100	100	100	1.000	1.000	1.000
Dressing changing times	3.47 ± 1.29	4.69 ± 1.03	1.60 ± 0.96	3.55 ± 1.35	4.55 ± 1.37	1.47 ± 0.95	0.471	0.431	1.034
Pain score on day 3	1.86 ± 1.06	2.31 ± 1.25	1.98 ± 0.83	2.15 ± 1.00	2.00 ± 0.89	1.89 ± 0.76	0.225	0.706	0.766
Pain score by last treatment	0.37 ± 0.57	0.42 ± 0.51	0.18 ± 0.45	0.43 ± 0.68	0.40 ± 0.52	0.04 ± 0.29	0.886	0.039	0.030
Pain score declining	1.49 ± 0.98	1.92 ± 0.95	1.80 ± 0.91	1.72 ± 0.93	1.64 ± 0.67	1.85 ± 0.75	0.301	0.925	0.579
Wound condition score before treatment	8.33 ± 1.61	9.62 ± 1.80	7.83 ± 1.69	8.68 ± 1.59	8.09 ± 1.64	7.98 ± 1.47	0.336	0.022	0.731
Wound condition score after treatment	4.00 ± 0.00	4.00 ± 0.00	4.00 ± 0.00	4.00 ± 0.00	4.00 ± 0.00	4.00 ± 0.00	1.000	1.000	1.000
Wound condition score improvement	4.33 ± 1.61	5.62 ± 1.80	3.83 ± 1.69	4.64 ± 1.57	4.09 ± 1.64	3.98 ± 1.47	0.379	0.022	0.731
Improvement in erythema and swelling	1.92 ± 0.76	2.08 ± 0.86	0.80 ± 0.65	1.87 ± 0.77	1.73 ± 0.79	0.85 ± 0.69	0.838	0.227	0.756
Improvement in exudate	1.96 ± 0.82	2.31 ± 0.63	1.63 ± 0.63	2.15 ± 0.75	2.09 ± 0.70	1.70 ± 0.59	0.267	0.457	0.498
Improvement in hemorrhage	0.35 ± 0.56	0.62 ± 0.65	1.35 ± 0.83	0.53 ± 0.65	0.09 ± 0.30	1.40 ± 0.65	0.142	0.025	0.717
Improvement in subeschar purulence and exudation	0.10 ± 0.31	0.62 ± 0.87	0.05 ± 0.22	0.09 ± 0.28	0.18 ± 0.40	0.02 ± 0.15	0.783	0.150	0.475
Drug treatment	40 (81.63)	13 (100.0)	37 (92.50)	44 (93.62)	11 (100.0)	47 (100.0)	0.076	1.00	0.093
Adverse event, *n* (%)	1 (2.04)	0 (0.00)	4 (10.00)	1 (2.13)	0 (0.00)	10 (21.28)	1.000	1.000	0.154

**Table 7:** Changes of wound conditions in 7 days of treatment.

Parameter	BC group			VG group			*p* value (BC versus VG)	
	Day 3	Day 7	*p* value	Day 3	Day 7	*p* value	Day 3	Day 7
Erythema and swelling	2.50 ± 0.92	1.30 ± 0.61	0.01	2.42 ± 0.90	1.31 ± 0.52	0.01	0.522	0.896
Exudation	2.87 ± 0.75	1.39 ± 0.66	0.01	2.94 ± 0.70	1.43 ± 0.68	0.01	0.489	0.696
Hemorrhage	1.77 ± 0.83	1.04 ± 0.20	0.01	1.88 ± 0.79	1.04 ± 0.19	0.01	0.369	0.967
Subeschar purulence and exudation	1.15 ± 0.43	1.08 ± 0.27	0.175	1.07 ± 0.25	1.07 ± 0.29	1.000	0.101	0.762
Pain score	1.96 ± 1.00	0.98 ± 0.99	0.01	2.02 ± 0.89	1.13 ± 0.87	0.01	0.659	0.239

## Data Availability

The datasets used and/or analyzed during the current study are available from the corresponding author upon reasonable request.
